The article "Polyethylene glycol-doped BiZn2VO6 as a high-efficiency solar-light-activated photocatalyst with substantial durability toward photodegradation of organic contaminations" was retracted in 2023. Reasons: an official misconduct investigation; misconduct by an author.

# Polyethylene glycol-doped BiZn_2_VO_6_ as a high-efficiency solar-light-activated photocatalyst with substantial durability toward photodegradation of organic contaminations

**DOI:** 10.1039/c8ra06896h

**Published:** 2018-11-07

**Authors:** Mahsa Pirhashemi, Sami Elhag, Aziz Habibi-Yangjeh, Galia Pozina, Magnus Willander, Omer Nur

**Affiliations:** Department of Science and Technology (ITN), Linköping University, Campus Norrköping SE-601 74 Norrköping Sweden mahsa.pirhashemi@liu.se mahsapirhashemi@uma.ac.ir; Department of Chemistry, Faculty of Science, University of Mohaghegh Ardabili P. O. Box 179 Ardabil Iran; Department of Physics, Chemistry and Biology (IFM), Linköping University S-581 83 Linköping Sweden

## Abstract

In this study, we focus on a simple, low-priced, and mild condition hydrothermal route to construct BiZn_2_VO_6_ nanocompounds (NCs) as a novel photocatalyst with strong solar light absorption ability for environmental purification using solar energy. NCs were further doped with polyethylene glycol (PEG) to improve their photocatalytic efficiency for photodegradation processes through inhibition of fast charge carrier recombination rates and higher charge separation efficiency. Surface morphology, phase structure, optical characteristics, and band structure of the as-prepared samples were analyzed using XRD, EDX, XPS, SEM, UV-vis spectroscopy, CL, and BET techniques. PEG-doped BiZn_2_VO_6_ NCs were applied as effective materials to degrade various kinds of organic pollutants including cationic and anionic types, and these NCs exhibited excellent photocatalytic efficiency as compared to traditional photocatalysts. In particular, the PEG-doped BiZn_2_VO_6_ (0.10% w/v) photocatalyst exhibited highly enhanced photocatalytic performance with improvements of about 46.4, 28.3, and 7.23 folds compared with PEG-doped ZnO nanorods (NRs), pristine BiVO_4_, and BiZn_2_VO_6_ samples, respectively, for the decomposition of congo red (CR) dye. After 40 minutes of sunlight irradiation, 97.4% of CR was decomposed. In this study, scavenging experiments indicated that both hydroxyl radicals and holes play dominant roles in CR photodegradation under simulated solar light irradiation. Meanwhile, the optimal photocatalyst demonstrated good reproducibility and stability for successive cycles of photocatalysis.

## Abstract 2

In this study, we focus on a simple, low-priced, and mild condition hydrothermal route to construct BiZn_2_VO_6_ nanocompounds (NCs) as a novel photocatalyst with strong solar light absorption ability for environmental purification.

## 1. Introduction

With rapid industrialization and increasing population, energy deficiency and environmental pollution have become increasingly drastic obstacles in recent years.^1,2^ In particular, industrial dyes are accountable for water-pollution, and these organic pollutants can produce hazardous compounds through hydrolysis, oxidation, or other chemical reactions in the wastewater.^3^ Therefore, the elimination of these poisonous organic compounds from wastewater with efficient methods remains a challenging task. One of the promising methods to overcome this obstacle is entire degradation of these aqueous contaminants using semiconductor-based photocatalysis utilizing solar energy under relatively mild operating conditions.^4^ As is well-known, utilization of the most widely studied and used photocatalysts such as TiO_2_ and ZnO is severely restricted because of their wide band gap energy (≥3.2 eV), which indicates that they perform poorly as photocatalysts under visible light. Regrettably, fast recombination of photo-induced charges in these semiconductors also limits their photocatalytic applications.^5,6^ In this field, studies are focused on the chemical modification of photocatalysts with wide band gap, aiming to alter the band gap or enhance the separation of electron–hole pairs; also, single-phase photocatalysts with satisfactory photocatalytic properties for the degradation of organic pollutants are developed, and they include g-C_3_N_4_,^7^ Bi_2_O_2_CO_3_,^8^ Bi_2_Ga_4_O_9_,^9^ and BiFeO_3_.^10^ Hence, robust and solar-responsive photocatalysts are urgently needed as the next-generation photocatalysts, which can provide favorable condition to use all wavelengths of sunlight.

The article "Polyethylene glycol-doped BiZn2VO6 as a high-efficiency solar-light-activated photocatalyst with substantial durability toward photodegradation of organic contaminations" was retracted in 2023. Reasons: an official misconduct investigation; misconduct by an author.

A novel type of mixed metal oxides represented by the main formula BiM_2_AO_6_ with M = Mg, Ca, Cd, Cu, Pb, Mn, and Zn and A = V, P, As has become a research focus as potential alternative semiconductors for sunlight-driven photocatalysts in recent years.^11–16^ These compounds have been examined broadly based on their luminescence, magnetic, and photocatalytic properties as well as nonlinear optical characteristics. Among these semiconductors, bismuth zinc vanadate (BiZn_2_VO_6_) is a promising material due to its outstanding properties: suitable band gap of 2.4 eV, low price, high chemical durability, and accessibility.^17–19^ For example, Nunes *et al.*^17^ reported a computational study based on density functional theory (DFT), which demonstrated that BiZn_2_VO_6_ has a unique crystal structure and electronic properties as a narrow band gap semiconductor. Luo *et al.*^20^ synthesized BiZn_2_VO_6_ ceramic by the solid state reaction method, which showed desirable microwave dielectric properties and also exhibited good sintering behavior such as great chemical compatibility with Ag electrodes at 780 °C grown for 4 h. In addition, BiZn_2_VO_6_ as a thin film electrode can also be applied for oxygen evolution applications due to its electrical and optical properties. For instance, Liu *et al.*^18^ presented that the photocurrents due to water oxidation at BiZn_2_VO_6_ particulate thin film electrodes can be efficiently enhanced by pre-treatment with an aqueous TiCl_4_ solution due to the facilitation of the transport of photogenerated electrons within BiZn_2_VO_6_ by the necking effect of the flock similar to a TiO_2_ overlayer. In another example, Liu *et al.*^19^ reported that BiZn_2_VO_6_ has a higher specific surface area compared to BiVO_4_ and exhibits excellent visible-light-driven photocatalytic O_2_ evolution efficiency; also, photoactivity can be remarkably increased by chemical etching with warm H_2_SO_4_.

The article "Polyethylene glycol-doped BiZn2VO6 as a high-efficiency solar-light-activated photocatalyst with substantial durability toward photodegradation of organic contaminations" was retracted in 2023. Reasons: an official misconduct investigation; misconduct by an author.

According to the interesting properties and high potential of BiZn_2_VO_6_ as a photocatalyst and to the best of our knowledge, no study has been conducted to investigate the photocatalytic activity of this unique semiconductor in the photodegradation of various organic dyes. However, a considerable impediment in employing this semiconductor as a solar-light-driven photocatalyst is the rapid recombination of its photo-generated e^−^/h^+^ pairs, resulting in poor performance. Among the various strategies employed to boost the overall photocatalytic efficiency,^21,22^ an interesting strategy to achieve a more efficient photocatalyst is the addition of organic agents as a dopant source.^23,24^ It has been reported that PEG is a polymeric material commonly used as a growth template for the synthesis of nanomaterials, and it can be employed to boost the morphology, specific surface area, and crystallographic properties of nanoparticles.^25–27^ Unlike the observations for many reports, in this study, PEG was used as a doping source, which could introduce a rich hydrogenated-environment around the synthesized photocatalysts. In this line, Zhang *et al.*^28^ demonstrated that water-soluble PEG has strong hydrogen bonding interactions between hydrogen in water and the hydroxyl oxygen in PEG, resulting in the disruption of hydrogen bonding when PEG dissolved in water provides a rich hydrogenated-environment for the growth of nanoparticles. In addition, theoretical as well as experimental studies have revealed a novel type of behavior for hydrogen as an impurity in semiconducting materials.^29–31^ It is generally acknowledged that hydrogen exhibits amphoteric effect, which indicates that it can play the role of a donor (H^+^) or an acceptor (H^−^) depending on the Fermi level of semiconductors.^32–35^ Consequently, this amphoteric behavior precludes hydrogen from acting as a dopant, *i.e.*, from being a source of conductivity. Based on first-principle calculation, van de Valle theoretically reported this feature of hydrogen in ZnO.^36^ Moreover, several experimental studies have confirmed that hydrogen improves electrical conductivity mainly by increasing the free carrier concentration and/or the carrier mobility.^37–40^ Also, it is beneficial for decreasing the recombination rate of the light-induced e^−^/h^+^ pairs and stabilizing the charge carriers on the surface of photocatalyst, eventually elevating the photocatalytic reaction efficiency. Adhering to this idea, several researchers have also obtained high photoconductivity and infrared absorption with hydrogen-related impurity in ZnO structures.^41–43^ Recently, our group reported the introduction of PEG as a hydrogen source in a ZnO NR structure, promoting elecro-catalytic properties and boosting the performance of ZnO NRs as a sensing electrode. In that study, Elhag *et al.* completely characterized and demonstrated enhanced optical and electronical properties of PEG-doped ZnO NRs with retention of morphology and structure.^44^ Most recently, Elhag *et al.* have also intensively investigated photoelectrochemical properties of PEG-doped BiZn_2_VO_6_ as a photoelectrode and demonstrated that PEG doping can enhance the charge collection efficiency and photocurrent density of BiZn_2_VO_6_ semiconductor.^32^

The article "Polyethylene glycol-doped BiZn2VO6 as a high-efficiency solar-light-activated photocatalyst with substantial durability toward photodegradation of organic contaminations" was retracted in 2023. Reasons: an official misconduct investigation; misconduct by an author.

Accordingly, the main aim of the present research is to study the photocatalytic degradation of various dyes that are extensively used by the textile industry in the presence of PEG-doped BiZn_2_VO_6_ as a suitable solar-light-activated photocatalyst. The synthesis of BiZn_2_VO_6_ semiconductor is mostly carried out under extreme conditions including long reaction duration and high temperature.^18–20^ Therefore, it is imperative to develop methods that are simple and fast for the fabrication of BiZn_2_VO_6_ photocatalysts that yield high photocatalytic activity and stability.

In the synthetic procedure applied here, we demonstrate an attempt to synthesize PEG-doped BiZn_2_VO_6_ NCs using PEG-doped ZnO nanorods (NRs) along with BiVO_4_ through a facile hydrothermal method. The novelty of this route lies in its simplicity, utilization of low temperature, and the capability of producing solar light-responsive photocatalysts by a quick and template-free approach. The photocatalytic performance of the as-fabricated photocatalysts was evaluated with respect to these processing conditions by kinetic analysis of various dye photodegradation experiments. The results were assessed to determine the photocatalytic performance of these remarkable solar-driven photocatalysts. Interestingly, our photodegradation efficiency towards cationic and anionic dyes is comparable to those of many recently reported metal oxide-based photocatalysts.^45–47^ The results of these experiments demonstrated enhanced photocatalytic ability. Due to relatively low cost and convenience, PEG-doped BiZn_2_VO_6_ NCs can be used as an available photocatalyst for the disposal of industrial effluents.

The article "Polyethylene glycol-doped BiZn2VO6 as a high-efficiency solar-light-activated photocatalyst with substantial durability toward photodegradation of organic contaminations" was retracted in 2023. Reasons: an official misconduct investigation; misconduct by an author.

## 2. Experimental details

### 2.1. Materials

All chemicals of analytical grade were obtained from Sigma-Aldrich, Germany, and were used without further purification. Also, deionized water was employed for all experiments.

### 2.2. Preparation of pristine and PEG-doped ZnO nanorods

Briefly, pristine and PEG-doped ZnO NRs were synthesized using a simple hydrothermal method, as reported previously.^44^ For the preparation of pristine ZnO NRs, 0.05 M aqueous solutions of Zn(NO_3_)_2_·6H_2_O and C_6_H_12_N_4_ were mixed. After magnetically stirring at room temperature, the homogenous solution was placed in an oven for 5 hours at 90 °C. Afterwards, the separated precipitates were washed with deionized water and acetone and then dried overnight at 60 °C. Upon adding 0.10% (w/v) PEG 2000, PEG-doped ZnO NRs were prepared by the same method as stated above.

### 2.3. Synthesis of PEG-doped BiZn_2_VO_6_ photocatalysts

In a typical synthetic route for the preparation of PEG-doped BiZn_2_VO_6_ (0.10% w/v), 0.10% (w/v) represents 0.10 g of PEG-doped ZnO. First, 0.02 M of Bi(NO_3_)_3_·5H_2_O and NH_4_VO_3_ were dissolved in 10 ml of nitric acid (70%) solution. Then, 20 ml deionized water was added to this solution with constant stirring until the salts were mixed properly. Thereafter, a certain amount of NaHCO_3_ was used to adjust the pH to ∼6.5 and an apparently homogeneous yellow solution was formed. Next, 0.10 g of the as-prepared PEG-doped ZnO NRs was dispersed into this yellow solution and then, the suspension was placed in a preheated oven for 4 hours at 80 °C. The resulting nanoparticles were rinsed with deionized water and acetone and then dried at 60 °C for 10 h in an oven. The same procedure was repeated for non-doped BiZn_2_VO_6_ with the exception of the addition of PEG. A schematic diagram for the fabrication of the photocatalyst is presented in Fig. 1.

**Fig. 1:** Schematic illustration for synthesis procedure of the PEG-doped BiZn_2_VO_6_ photocatalysts.

### 2.4. Characterization instruments

X-ray power diffraction (XRD) patterns ranging from 10° to 70° of the as-synthesized samples were provided using a Philips PW 1729 with Cu Kα radiation source. Scanning electron microscopy (SEM) observations were performed by means of a LEO 1550 Gemini field emission gun at 5 kV. Purity and elemental analysis of the photocatalyst were obtained by EDX at 20 kV on the same SEM instrument. Defect analysis was performed using cathodoluminescence (CL) on a Gatan MonoCL4 system combined with the SEM apparatus. Also, X-ray photoelectron spectroscopy (XPS) data were captured on a Scienta ESCA200 spectrometer with Al Kα radiation. The binding energies were fitted by employing C 1s of adventitious carbon (284.8 eV) as a reference. N_2_ gas sorption analysis of the photocatalysts was performed on a Belsorp mini II apparatus at 77 K. Fourier transform-infrared (FTIR) spectra were recorded using a Perkin Elmer Spectrum RX I. Optical properties of the samples were conducted using a UV-visible spectrophotometer on a PerkinElmer Lambda 900 apparatus.

The article "Polyethylene glycol-doped BiZn2VO6 as a high-efficiency solar-light-activated photocatalyst with substantial durability toward photodegradation of organic contaminations" was retracted in 2023. Reasons: an official misconduct investigation; misconduct by an author.

### 2.5. Photocatalytic tests

The photocatalytic performances of the prepared samples were measured by photodegradation of 20 mg l^−1^ congo red (CR), methylene blue (MB), and rhodamine b (RhB) solutions as pollutants. The light source was a 300 W xenon lamp used without any filter to simulate sunlight irradiation. First, 50 mg of the photocatalyst was dispersed in 100 ml of the dye solution; the suspension was stirred in dark for 30 minutes to obtain adsorption–desorption equilibrium between the photocatalyst and the dye molecules prior to exposure to light. After the lamp was turned on, the samples were taken in specific desired time intervals within 90 minutes of the reaction time. The change in the concentration of the dye solution was evaluated using UV-vis absorption spectroscopy at characteristic absorption wavelengths of 497, 664, and 553 nm for CR, MB, and RhB, respectively.

## 3. Results and discussion

### 3.1. Morphological and structural characterization of the photocatalysts

XRD evaluation was performed to investigate the crystal structures and phase purities of the samples of ZnO NRs, PEG-doped ZnO NRs, BiVO_4_, BiZn_2_VO_6_, and PEG-doped BiZn_2_VO_6_; the patterns are illustrated in Fig. 2. Compared with the typical diffraction peak of standard ZnO (JCPDS no. 36-1451), ZnO NRs with and without PEG were suggested to be hexagonal wurtzite phase ZnO.^48^ In addition, the XRD pattern of BiVO_4_ showed good agreement with the reference card (JCPDS no. 74-4894) corresponding to the monoclinic phase of BiVO_4_.^49^ With respect to the BiZn_2_VO_6_ sample, the diffraction peaks at 23.5°, 28.9°, 31.6°, 34.2°, 36.9°, 39.1°, 46.6°, and 48.5° were indexed to (101), (103), (110), (006), (105), (114), (200), and (116) planes, respectively, of orthorhombic BiZn_2_VO_6_ (JCPDS no. 01-075-9214).^50^ The above results demonstrate that PEG-doped BiZn_2_VO_6_ samples are successfully obtained, and the crystalline phase of BiZn_2_VO_6_ is not affected seriously after loading of PEG. Besides, no additional crystal phases or impurities were observed, implying that the as-synthesized samples are unadulterated.

The article "Polyethylene glycol-doped BiZn2VO6 as a high-efficiency solar-light-activated photocatalyst with substantial durability toward photodegradation of organic contaminations" was retracted in 2023. Reasons: an official misconduct investigation; misconduct by an author.

**Fig. 2:** XRD patterns for ZnO NRs, PEG-doped ZnO NRs, BiVO_4_, BiZn_2_VO_6_, and PEG-doped BiZn_2_VO_6_ with different (w/v) percentages of PEG.

Elemental analysis has been performed to verify the chemical constituents of PEG-doped BiZn_2_VO_6_ (0.10% w/v) sample using spot EDX analysis (Fig. 3a). Except for some Au peaks of the substrate, EDX spectrum indicates that the sample contains only Bi, Zn, V, and O, confirming high degree of purity of the as-prepared PEG-doped BiZn_2_VO_6_ (0.10% w/v) sample. Additionally, EDX mappings are performed to investigate the elemental distribution of PEG-doped BiZn_2_VO_6_ (0.10% w/v), and the results are presented in Fig. 3b–g. It can be observed that Bi, Zn, V, and O are uniformly distributed over the whole sample area.

**Fig. 3:** (a) EDX spectrum and (b–g) EDX mapping for PEG-doped BiZn_2_VO_6_ (0.10% w/v) sample.

Morphologies of the synthesized samples are further investigated through SEM images, as depicted in Fig. 4. It is clear that the ZnO sample presents uniform nanorod morphology. The ZnO nanorod particles are formed with the hexagonal wurtzite structure with diameters of around 400 nm and lengths of up to several micrometers. Furthermore, the PEG-doped ZnO sample (Fig. 4b) exhibits the same features with slightly smaller diameters than that of ZnO NRs. The widths of these PEG-doped ZnO NRs are between 250 nm and 300 nm with length of about one micrometer. In addition, the BiVO_4_ nanocrystals indicate a spherical configuration (Fig. 4c) and are composed of numerous BiVO_4_ sub-nanoparticles; also, the degree of agglomeration is high. Interestingly, after introducing PEG-doped ZnO NRs in the BiVO_4_ environment, due to strong interactions and etching effect on the nanorods in the growth solution at pH ∼6.5, the BiZn_2_VO_6_ particles start to grow and exhibit notable changes in size and features compared with pristine ZnO NRs and BiVO_4_ samples (Fig. 4d). As clearly seen from the SEM image of the PEG-doped BiZn_2_VO_6_ (0.10% w/v) sample, it has aggregated structures of large-sized and denser particles.

**Fig. 4:** SEM images of (a) ZnO NRs, (b) PEG-doped ZnO NRs, (c) BiVO_4_, and (d) PEG-doped BiZn_2_VO_6_ (0.10% w/v) samples.

Surface-sensitive XPS analysis further confirms the composition and valence states of the constituent elements of the PEG-doped BiZn_2_VO_6_ (0.10% w/v) photocatalyst. The survey XPS spectrum (Fig. 5a) of the PEG-doped BiZn_2_VO_6_ (0.10% w/v) sample exhibits peaks corresponding to Bi 4f, Zn 2p, V 2p, O 1s, and C 1s without any impurities. Zn 2p high resolution XPS spectrum in Fig. 5b exhibits binding energies of Zn 2p_3/2_ and Zn 2p_1/2_ at 1022.4 and 1045.2 eV, respectively, which are an indication of the presence of Zn^2+^ in PEG-doped BiZn_2_VO_6_ (0.10% w/v).^51^ As shown in Fig. 5c, there are two intense peaks at 159.0 eV and 164.4 eV for the PEG-doped BiZn_2_VO_6_ (0.10% w/v) photocatalyst, which are ascribed to Bi 4f_7/2_ and Bi 4f_5/2_ and correspond to Bi^3+^.^52,53^ Also, the XPS data for pristine BiVO_4_ are shown in Fig. 5c for comparison. The binding energies of Bi 3f_7/2_ and Bi 3f_5/2_, at 159.8 and 165.1 eV, respectively, for pristine BiVO_4_ are slightly lower than those for Bi in the PEG-doped BiZn_2_VO_6_ (0.10% w/v) material. Moreover, Fig. 5d provides the spectrum for V 2p. For PEG-doped BiZn_2_VO_6_ (0.10% w/v), the peak at 517.0 eV is ascribed to V 2p_3/2_ and the other peak at 525.1 eV belongs to V 2p_1/2_, which are characteristics of V^5+^ ions. Compared with the results for pristine BiVO_4_, a shift of 0.5 eV is observed in the peak position corresponding to V 2p (516.5 for V 2p_3/2_ orbital and 524.6 eV for V 2p_1/2_).^54^ In the XPS spectrum for O 1s (Fig. 5e), one characteristic peak at 532.1 eV and a shoulder at 530 eV are clearly detected, which are in agreement with the results for lattice oxygen and oxygen species of hydroxyl groups adsorbed on the surface, respectively.^32^ It is noticeable that the peak of O–H in PEG-doped BiZn_2_VO_6_ (0.10% w/v) is stronger than that of BiVO_4_, which demonstrates that the hydroxyl content in PEG-doped BiZn_2_VO_6_ is higher than that on BiVO_4_. Generally, more hydroxyl contents on the surface of a photocatalyst have a positive effect on photocatalytic proficiency.^35^ This can be further confirmed by the results obtained from photocatalytic performance. Consequently, the peak shifts (increase in binding energy of Bi 4f and V 2p in PEG-doped BiZn_2_VO_6_ (0.10% w/v)) are in fact due to the incorporation of ZnO components into the BiVO_4_ structure and chemical interactions between the material components, which lead to the growth of mixed metal oxide semiconductor, as previously reported.^32^ Therefore, XPS results demonstrated successful fabrication of PEG-doped BiZn_2_VO_6_ photocatalyst.

The article "Polyethylene glycol-doped BiZn2VO6 as a high-efficiency solar-light-activated photocatalyst with substantial durability toward photodegradation of organic contaminations" was retracted in 2023. Reasons: an official misconduct investigation; misconduct by an author.

**Fig. 5:** XPS spectra for the PEG-doped BiZn_2_VO_6_ (0.10% w/v): (a) survey scan and high-resolution spectra for: (b) Zn 2p, (c) Bi 4f, (d) V 2p, and (e) O 1s compared with pristine BiVO_4_ nanoparticles.

UV-vis absorption spectroscopy was applied to investigate the optical properties of the samples. In general, the light-harvesting efficiencies for photocatalysts are of vital importance for their applications in the degradation of organic dyes.^55^ As expected from a wide band gap semiconductor, it is clear that ZnO NRs only absorb UV light, whereas according to literatures, PEG-doped ZnO NRs show small red-shift in the absorption edge.^44,56^ However, as seen in Fig. 6, the BiVO_4_ sample clearly exhibits enhanced absorption in the UV-visible region. It is also clear that PEG-doped BiZn_2_VO_6_ (0.10% w/v) exhibits clear absorbance in UV and visible regions. Accordingly, improved light-harvesting ability of the photocatalyst can boost light utilization and consequently enhance its photocatalytic performance.

**Fig. 6:** UV-vis absorption spectra for BiVO_4_ and PEG-doped BiZn_2_VO_6_ (0.10% w/v) samples.

The CL technique is also a beneficial method for determining the optical properties of nanostructures.^57^ Besides, CL uses a high-energy electron beam for excitation and all CL spectra are measured at room temperature. Due to the polycrystalline nature of PEG-doped BiZn_2_VO_6_ (0.10% w/v) photocatalyst, uniformity of the electronic characteristics of different points on the surface was investigated by CL and the results are illustrated in Fig. 7. The measured CL spectra of the as-prepared PEG-doped BiZn_2_VO_6_ (0.10% w/v) sample at three points are quite similar, suggesting isotropic electronic features of the sample. Furthermore, the results exhibit an evident luminescence band between 540 and 610 nm, which is ascribed to deep level emission (450–660 nm),^58^ demonstrating the presence of interstitial oxygen (O_i_) or hydroxyl groups on the surface of the photocatalyst. As a result, green emission is caused from the recombination between holes trapped at the surface defects and electrons trapped at the oxygen vacancies, which can boost photocatalytic activity by reducing the recombination rate of e^−^/h^+^ pairs.^59,60^

**Fig. 7:** CL spectra of PEG-doped BiZn_2_VO_6_ (0.10% w/v). The inset shows an SEM image of the sample, where the numbers correspond to the locations of CL measurements.

### 3.2. Evaluation of photocatalytic performance

It is important to note that CR was selected as the typical resistant dye to estimate the photocatalytic performance of obtained photocatalysts. Fig. 8a shows the degradation efficiencies of CR with different photocatalysts. As observed, there is no distinct CR degradation in the presence of simulated solar light without any photocatalyst, indicating high stability of CR under light illumination. In addition, pure ZnO NRs and BiVO_4_ illustrated low photocatalytic degradation efficiencies of approximately 11.9% and 23.1%, respectively, in 90 min of light irradiation. This is related to the rapid recombination of e^−^/h^+^ pairs in these semiconductors although BiVO_4_ can strongly absorb visible light due to narrow band-gap energy. However, as a key result, the addition of PEG to ZnO NRs caused 14.6% increase in CR degradation in comparison with that for the pure ZnO NR photocatalyst. Also, the relative photodegradation efficiency of PEG-doped BiZn_2_VO_6_ photocatalyst presented crucial improvements in contrast to that of pure BiZn_2_VO_6_. This confirmed that the presence of PEG influenced the photocatalytic activity of the photocatalyst. Besides, the highest removal efficiency of CR reached 97.4% for the prepared PEG-doped BiZn_2_VO_6_ (0.10% w/v) sample within 40 min under simulated solar light irradiation. Clearly, the introduction of PEG enhanced the photocatalytic degradation ability of BiZn_2_VO_6_; however, the content of PEG exhibited serious impact on the proficiency of photocatalysts and 0.10% (w/v) of PEG was determined as the optimal amount. As a result, the synergistic effect of PEG and BiZn_2_VO_6_ appreciably promoted the separation of the photo-induced e^−^/h^+^ pairs, which has a beneficial effect on the photocatalytic reactions. Such a phenomenon has been previously proved by photoluminescence and photocurrent measurements reported by Elhag *et al.*^32^

The article "Polyethylene glycol-doped BiZn2VO6 as a high-efficiency solar-light-activated photocatalyst with substantial durability toward photodegradation of organic contaminations" was retracted in 2023. Reasons: an official misconduct investigation; misconduct by an author.

**Fig. 8:** (a) Photodegradation of CR over ZnO NRs, BiVO_4_, PEG-doped ZnO NRs, BiZn_2_VO_6_, and PEG-doped BiZn_2_VO_6_ NCs with different (w/v) percentages of PEG. UV-vis spectra for degradation of CR under solar simulated light irradiation over (b) PEG-doped ZnO NRs, (c) BiVO_4_, (d) BiZn_2_VO_6_, and (e) PEG-doped BiZn_2_VO_6_ (0.10% w/v) photocatalysts.

Changes in UV-vis absorbance spectra of CR as a function of irradiation time in the presence of PEG-doped ZnO NR, BiVO_4_, BiZn_2_VO_6_, and PEG-doped BiZn_2_VO_6_ (0.10% w/v) samples are shown in Fig. 8b–e. Evidently, the characteristic absorption peak of CR diminishes slightly over PEG-doped ZnO NR, BiVO_4_, and BiZn_2_VO_6_ samples with prolonged light illumination time. However, as shown in Fig. 8e, the intensity of the major peak rapidly weakens and becomes stable, indicating that the CR structure is successfully degraded by PEG-doped BiZn_2_VO_6_ (0.10% w/v) photocatalyst. Additionally, the degradation efficiency of our present photocatalytic system is compared with those of other recently reported photocatalysts for the photocatalytic degradation of CR, and the results are summarized in Table 1.^61–66^ The results demonstrate that PEG-doped BiZn_2_VO_6_ (0.10% w/v) is a better photocatalyst with respect to the duration of reaction and degradation efficiency.

The article "Polyethylene glycol-doped BiZn2VO6 as a high-efficiency solar-light-activated photocatalyst with substantial durability toward photodegradation of organic contaminations" was retracted in 2023. Reasons: an official misconduct investigation; misconduct by an author.

**Table 1:** Comparison of CR photodegradation efficiency over different photocatalysts

Photocatalyst	Light source	CR concentration	Photocatalyst amount	Photodegradation efficiency	Ref.
Mesoporous sphere-like Cu_2_O	Xe 300 W	1.4 × 10^−5^ M	50 mg	97% in 90 min	61
BiFeO_3_/N-doped graphene	Xe 300 W (UV cut-off filter)	10 mg l^−1^	0.02 g	55% in 120 min	62
ZnO/ZrO_2_	UV 15 W	10 ppm	0.05 g	90% in 120 min	63
α-MnO_2_	500 W halogen lamp	40 mg l^−1^	0.10 g	>90% in 70 min	64
ZnAl_2_O_4_ nanoparticles	500 W mercury lamp	15 mg l^−1^	50 mg	98.3% in 80 min	65
BiOCl–Ag_8_SnS_6_	Sunlight radiation	20 mg l^−1^	100 mg	>99% in 90 min	66
PEG-doped BiZn_2_VO_6_ (0.10% w/v)	Xe 300 W	20 mg l^−1^	50 mg	>99% in 40 min	This work

To quantitatively evaluate the photocatalytic performance of the samples, the observed first-order rate constants (*k*_obs_) of different photocatalysts were obtained according to a pseudo-first-order kinetic model.^67,68^ The calculated rate constants are presented in Fig. 9. All as-prepared PEG-doped BiZn_2_VO_6_ samples showed an abrupt increase in CR degradation under the stated conditions. The degradation rate constant of CR over PEG-doped BiZn_2_VO_6_ (0.10% w/v) was calculated to be 831 × 10^−4^ min^−1^, which is about 46.4, 28.3, and 7.23 times higher than those of PEG-doped ZnO NRs (17.3 × 10^−4^ min^−1^), BiVO_4_ (29.4 × 10^−4^ min^−1^), BiZn_2_VO_6_ (115 × 10^−4^ min^−1^), respectively. The origin of superior photocatalytic performance of the PEG-doped BiZn_2_VO_6_ (0.10% w/v) photocatalyst can be ascribed to efficient separation and rapid transfer of photo-induced e^−^/h^+^ as well as relatively higher light absorption ability of the photocatalyst.

**Fig. 9:** The degradation rate constants of CR over ZnO NRs, PEG-doped ZnO NRs, BiVO_4_, BiZn_2_VO_6_, and PEG-doped BiZn_2_VO_6_ NCs with different (w/v) percentages of PEG.

As an important influencing factor of photocatalytic performance, Brunauer–Emmett–Teller (BET) specific surface areas of samples were measured by the N_2_ adsorption/desorption BET method, and the results are presented in Fig. 10. Furthermore, the BET surface areas of samples, calculated using the N_2_ adsorption/desorption isotherm data, are presented in Table 2 together with the mean pore diameters and total pore volumes. It is evident that all curves exhibit small H1-type hysteresis loops, which are ascribed to type IV isotherms and are representative of mesoporous materials.^69^ The BET specific surface area of PEG-doped ZnO NRs is 10.5 m^2^ g^−1^, which is about 4.8 times higher than that of pristine ZnO NRs (2.22 m^2^ g^−1^). This indicates that doping PEG is a feasible method to increase the BET surface area of the host. It is clear that the surface area, mean pore diameter, and total pore volume of PEG-doped BiZn_2_VO_6_ NCs are greater than those of the PEG-doped ZnO NR and BiVO_4_ samples. Thus, because of their large textural properties, PEG-doped BiZn_2_VO_6_ NCs provide more photocatalytic reaction sites for the adsorption of reactant molecules and capture of the irradiation light. This also increases the efficiency of e^−^/h^+^ separation;^46^ thus, the photocatalytic activity of PEG-doped BiZn_2_VO_6_ NCs is enhanced. Among all samples, the PEG-doped BiZn_2_VO_6_ (0.15% w/v) photocatalyst has the largest specific surface area. However, its photocatalytic activity is lower than that of the PEG-doped BiZn_2_VO_6_ (0.10% w/v) photocatalyst, which can be related to the efficient separation of charge carriers in the PEG-doped BiZn_2_VO_6_ (0.10% w/v) photocatalyst in comparison to that in the PEG-doped BiZn_2_VO_6_ (0.15% w/v) photocatalyst. Therefore, appropriate loading of PEG is important for achieving the best photocatalytic performance.

The article "Polyethylene glycol-doped BiZn2VO6 as a high-efficiency solar-light-activated photocatalyst with substantial durability toward photodegradation of organic contaminations" was retracted in 2023. Reasons: an official misconduct investigation; misconduct by an author.

**Fig. 10:** Nitrogen gas adsorption–desorption data over ZnO NRs, PEG-doped ZnO NRs, BiVO_4_, and PEG-doped BiZn_2_VO_6_ NCs with different (w/v) percentages of PEG.

**Table 2:** Texture properties of ZnO NRs, PEG-doped ZnO NRs, BiVO_4_, and PEG-doped BiZn_2_VO_6_ NCs with different (w/v) percentages of PEG

Photocatalyst	Surface area (m^2^ g^−1^)	Mean pore diameter (nm)	Total pore volume (cm^3^ g^−1^)
ZnO NRs	2.22	5.31	0.0049
PEG doped ZnO NRs	10.5	8.77	0.0139
BiVO_4_	3.59	5.46	0.0067
PEG-doped BiZn_2_VO_6_ (0.01% w/v)	9.29	5.68	0.0142
PEG-doped BiZn_2_VO_6_ (0.05% w/v)	10.4	11.9	0.0311
PEG-doped BiZn_2_VO_6_ (0.10% w/v)	12.8	13.1	0.0439
PEG-doped BiZn_2_VO_6_ (0.15% w/v)	20.8	13.7	0.0679

The well-known oxidative species in photocatalysis are photo-generated holes (h^+^) and free radicals such as superoxide radicals (˙O_2_^−^) and hydroxyl radicals (˙OH). To further identify the predominant active species for CR degradation over the PEG-doped BiZn_2_VO_6_ (0.10% w/v) photocatalyst in the reaction system, three typical scavengers, namely, 2-propanol (2-PrOH, 1 mM), ethylenediamintetraacetic acid (EDTA, 1 mM), and *p*-benzoquinone (BQ, 1 mM) were used for the estimation of the roles of ˙OH, h^+^, and ˙O_2_^−^, respectively. Reaction kinetic constants for processes with and without the relevant scavengers were examined, and the results are shown in Fig. 11. Clearly, all scavengers could partially suppress the photocatalytic efficiency of the optimal photocatalyst. However, the degradation rate constant of CR was slightly reduced after the addition of BQ, implying that only a few ˙O_2_^−^ species are produced in the degradation process. Conversely, in the presence of 2-PrOH and EDTA, the degradation rate constant of RhB was markedly restrained. Therefore, it can be inferred that ˙OH and h^+^ are the critical and responsible active species generated in the photodegradation process.

The article "Polyethylene glycol-doped BiZn2VO6 as a high-efficiency solar-light-activated photocatalyst with substantial durability toward photodegradation of organic contaminations" was retracted in 2023. Reasons: an official misconduct investigation; misconduct by an author.

**Fig. 11:** The degradation rate constants of CR over PEG-doped BiZn_2_VO_6_ (0.10% w/v) photocatalyst in the presence of different scavengers.

On the basis of the above experimental results and discussion, a suggested mechanism for the enhanced photoactivity of PEG-doped BiZn_2_VO_6_ photocatalysts is schematically presented in Fig. 12. The band edge positions of the conduction band (CB) and valence band (VB) of semiconductors can be calculated according to the Mulliken electronegativity theory:^70^

1 *E*_VB_ = *X* − *E*_e_ + 0.5*E*_g_

2 *E*_CB_ = *E*_VB_ − *E*_g_

Here, *X* is the absolute electronegativity of the semiconductor, and the *X* value for BiZn_2_VO_6_ is 5.81; *E*_e_ is the energy of free electrons on the hydrogen scale (about 4.5 eV), and *E*_g_ is the band gap of the semiconductor. The estimated VB and CB potentials are +0.3 and +2.7 eV, respectively, for BiZn_2_VO_6_. In the presence of solar simulated irradiation, the PEG-doped BiZn_2_VO_6_ NC photocatalyst absorbs photons and creates excited photo-electrons in CB and holes in VB of the semiconductor. Subsequently, PEG impurities can be regarded as active hydrogen-related defects that can act as shallow donors and enhance n-type conductivity of the photocatalyst, as has been proven in our previous study.^32^ In particular, the Mott–Schottky measurement confirms that hydrogen incorporated into BiZn_2_VO_6_ by PEG doping causes a shift in the Fermi level of PEG-doped BiZn_2_VO_6_ towards the conduction band edge in comparison with that observed for un-doped BiZn_2_VO_6_.^32^ These results are also consistent with previously published results by Cooper *et al.*,^71^ where they have reported an enhancement in n-type conductivity of BiVO_4_ due to hydrogen treatment. In addition, in our pervious study,^32^ based on the observed photocurrent and photoluminescence analysis, we showed that PEG modification can affect the separation efficiency of photo-generated electron/hole pairs. This is understood because the coverage of the nanoparticles by PEG molecules is due to intermolecular hydrogen bonds. Moreover, this result is also in agreement with the result of a recent study by Wang *et al.*^72^ Thus, doping of PEG introduces hydrogen impurities that act as effective shallow donors in BiZn_2_VO_6_ semiconductors; also, they play a vital role in the achieved conductivity and stabilize the photo-generated electrons and holes on the surface of as-prepared photocatalysts, leading to increased lifetime of the charge carriers. This consequently enhances their chance to reach the photocatalyst's surface to initiate photocatalytic reactions. Ultimately, the electrons generated in PEG-doped BiZn_2_VO_6_ NCs can further react with resolved O_2_ and H^+^ to produce H_2_O_2_, which can be further reduced to ˙OH radicals.^73^ Besides, VB of BiZn_2_VO_6_ edge is more positive than the standard redox potentials of ˙OH/H_2_O (+2.4 eV *vs.* NHE) and ˙OH/OH^−^ (+1.9 eV *vs.* NHE); thus, the photo-induced holes in VB can oxidize adsorbed H_2_O or OH^−^ molecules to ˙OH.^74,75^ Meanwhile, the VB holes are oxidative species and they can also eliminate organic pollutant molecules. Consequently, PEG-doped BiZn_2_VO_6_ NCs have high charge separation and transfer efficiency; when separated charge carriers react with surrounding water molecules, many reactive oxygen species are produced, which can effectively decompose the surrounding pollutant molecules.

The article "Polyethylene glycol-doped BiZn2VO6 as a high-efficiency solar-light-activated photocatalyst with substantial durability toward photodegradation of organic contaminations" was retracted in 2023. Reasons: an official misconduct investigation; misconduct by an author.

**Fig. 12:** A plausible diagram for separation of electron–hole pairs in the PEG-doped BiZn_2_VO_6_ photocatalysts.

The recyclability and stability are important factors for practical applications of photocatalysts. For this purpose, circulating experiments for the photodegradation of CR were performed to explore the stability of PEG-doped BiZn_2_VO_6_ (0.10% w/v) as a photocatalyst under simulated sunlight irradiation. Fig. 13a reveals that after four successive recycles, the photocatalyst only exhibited a marginal loss of its photocatalytic performance. A comparison of the XRD patterns and FT-IR spectra of the photocatalyst before and after four photocatalytic degradation cycles is presented in Fig. 13(b and c). No apparent changes are found before and after the cycling experiments, suggesting that the structure of PEG-doped BiZn_2_VO_6_ (0.10% w/v) photocatalyst does not change during the photocatalytic process. Hence, it is confirmed that the photocatalyst is not corroded during light irradiation and has excellent durability after multiple uses for photocatalytic degradation of pollutants in the liquid phase.

**Fig. 13:** (a) Reusability of the PEG-doped BiZn_2_VO_6_ (0.10% w/v) photocatalyst; (b and c) XRD patterns and Ft-IR spectra of the photocatalyst before and after four successive runs.

In addition, we studied the photocatalytic performance for the degradation of two more organic dyes (MB and RhB as cationic dyes) as probe reactions and demonstrated the enhancement in activity for PEG-doped BiZn_2_VO_6_ in comparison with that for PEG-doped ZnO NRs and BiVO_4_; the results are presented in Fig. 14. According to Fig. 8, similar to CR (as an anionic dye), RhB and MB dye solutions (as cationic dyes) showed no degradation without the photocatalyst under light illumination. As can be observed, the calculated RhB degradation rate constants were 35.7 × 10^−4^, 32.5 × 10^−4^ and 549 × 10^−4^ min^−1^ over PEG-doped ZnO NR, BiVO_4_ and PEG-doped BiZn_2_VO_6_ (0.10% w/v) photocatalysts, respectively. These results indicated that PEG-doped BiZn_2_VO_6_ exhibited a higher degradation rate constant compared to other photocatalysts, and indeed the enhanced activity of this photocatalyst was 15.4 and 16.9-folds better than those of PEG-doped ZnO NR and BiVO_4_ samples, respectively, for the degradation of RhB. Furthermore, the PEG-doped BiZn_2_VO_6_ photocatalyst showed maximal reaction rate constant for MB degradation (300 × 10^−4^ min^−1^), which was about 12.7 and 10.3 times superior than those of PEG-doped ZnO NRs (23.6 × 10^−4^ min^−1^) and BiVO_4_ (29.1 × 10^−4^ min^−1^), respectively. Hence, it can be concluded that the high activity profile of this photocatalyst for both cationic and anionic dyes makes it suitable for industrial wastewater treatment.

The article "Polyethylene glycol-doped BiZn2VO6 as a high-efficiency solar-light-activated photocatalyst with substantial durability toward photodegradation of organic contaminations" was retracted in 2023. Reasons: an official misconduct investigation; misconduct by an author.

**Fig. 14:** The degradation rate constants of CR, RhB, and MB over the PEG-doped ZnO NR, BiVO_4_, and PEG-doped BiZn_2_VO_6_ (0.10% w/v) samples under solar simulated light irradiation.

Finally, the photocatalytic activity of the PEG-doped BiZn_2_VO_6_ (0.10% w/v) photocatalyst was compared with those of other recently prepared photocatalysts, and the results are displayed in Table 3. As can be seen, compared to some of the reported visible-light-driven photocatalysts used in the photocatalytic degradation such as Bi_2_O_2_CO_3_ microspheres,^76^ Bi_2_Fe_4_O_9_/graphene,^77^ CeO_2_/Bi_2_MoO_6_,^78^ Bi_2_O_3_/g-C_3_N_4_ composite,^79^ and BiOBr/TiO_2_ nanofibers,^80^ PEG-doped BiZn_2_VO_6_ (0.10% w/v) exhibited better photodegradation effect for some organic dyes.^81^ In addition, PEG-doped BiZn_2_VO_6_ (0.10% w/v) presented enhanced activity in a shorter photodegradation time relative to other solar light-driven photocatalysts such as porphyrin-decorated Bi_2_O_2_CO_3_,^82^ BiOCl/Bi_2_Ti_2_O_7_,^83^ PEG-BiOCl,^84^ and MoS_2_–FeZnO.^85^ This verified that it can be categorized as one of the most active photocatalysts for the removal of various dyes.

**Table 3:** Comparison of photodegradation performances of PEG-doped BiZn_2_VO_6_ (0.10% w/v) with some reported photocatalysts^a^

Photocatalyst	Experimental conditions	Light source	Photodegradation efficiency (%)
Bi_2_O_2_CO_3_ microspheres	Catalyst = 0.01 g, [MO*] = 10 mg l^−1^, 100 ml	300 W Xe* lamp, *λ* ≥ 420 nm	98% in 180 min
Bi_2_Fe_4_O_9_/graphene	Catalyst = 30 mg, [MV*] = 30 mg l^−1^, 50 ml	Visible light irradiation	95% in 180 min
CeO_2_/Bi_2_MoO_6_	Catalyst = 50 mg, [RhB] = 10 mg l^−1^, [TC*] = 20 mg l^−1^, 100 ml	300 W Xe lamp, *λ* ≥ 400 nm	About 100% in 75 min, 78.7% in 120 min
Bi_2_O_3_/g-C_3_N_4_ composite	Catalyst = 20 mg, [AB 10B*] = 10 mg l^−1^, 50 ml	35 W Xe lamp	88.7% in 120 min
BiOBr/TiO_2_ nanofibers	Catalyst = 0.025 g, [4-NP*] = 10 mg l^−1^, 50 ml	250 W Xe lamp, *λ* ≥ 400 nm	About 100% in 180 min
Porphyrin-decorated Bi_2_O_2_CO_3_	Catalyst = 50 mg, [RhB*] = 0.5 mM, 50 ml, pH = 7.0	350 W Xe lamp	About 100% in 90 min
BiOCl/Bi_2_Ti_2_O_7_	Catalyst = 100 mg, [TC-HCl*] = 50 mg l^−1^, 100 ml	300 W Xe lamp	90% in 120 min
PEG–BiOCl	Catalyst = 15 mg, [MO] = 10 mg l^−1^, 50 ml, pH = 7.0	500 W Xe lamp	About 100% in 20 h
MoS_2_–FeZnO	Catalyst = 1 g l^−1^, [MB*] = 20 mg l^−1^, 150 ml	400 W halogen lamp	95% in 140 min
PEG doped BiZn_2_VO_6_ (this work)	Catalyst = 50 mg, [CR*] = 20 mg l^−1^, [RhB] = 20 mg l^−1^, [MB] = 20 mg l^−1^, 100 ml	300 W Xe lamp	97.4% in 40 min, 97.7% in 60 min, 96.1% in 100 min

a [*]: Xe = xenon, MO = methyl orange, RhB = rhodamine B, MV = methyl violet, TC = tetracycline, TC-HCl = tetracycline hydrochloride, AB 10B = amido black 10B, 4-NP = 4-nitrophenol, MB = methylene blue, CR = congo red.

The article "Polyethylene glycol-doped BiZn2VO6 as a high-efficiency solar-light-activated photocatalyst with substantial durability toward photodegradation of organic contaminations" was retracted in 2023. Reasons: an official misconduct investigation; misconduct by an author.

## 4. Conclusions

To sum up, a simple low-temperature hydrothermal method was applied to synthesize solar-light-activated PEG-doped BiZn_2_VO_6_ photocatalysts using PEG-doped ZnO NRs and pristine BiVO_4_ as starting materials. The as-prepared PEG-doped BiZn_2_VO_6_ NCs exhibited remarkably higher photocatalytic activities toward degradation of CR compared to PEG-doped ZnO NRs and pristine BiVO_4_. Photocatalytic processes of RhB and MB decomposition were also investigated. The PEG-doped BiZn_2_VO_6_ (0.10% w/v) photocatalyst exhibited the highest photo-activity, and the degradation efficiencies of CR, RhB, and MB were 97.4%, 97.6%, and 96.0%, respectively, which were much higher than those of PEG-doped ZnO NRs and pristine BiVO_4_. This distinctively enhanced photocatalytic activity of the PEG-doped BiZn_2_VO_6_ (0.10% w/v) photocatalyst was ascribed to its increased absorption of visible-light and higher efficiency in the separation and transfer of photo-induced electrons and holes. Furthermore, trapping experiments demonstrated that the main reactive species are ˙OH and h^+^ rather than ˙O_2_^−^. As a result, it can be deduced that this study can be useful to prepare more progressive and promising photocatalysts for environmental remediation and other industrial utilizations.

## Conflicts of interest

There are no conflicts to declare.

The article "Polyethylene glycol-doped BiZn2VO6 as a high-efficiency solar-light-activated photocatalyst with substantial durability toward photodegradation of organic contaminations" was retracted in 2023. Reasons: an official misconduct investigation; misconduct by an author.

## Supplementary Material

## References

[cit1] Holkar C. R., Jadhav A. J., Pinjari D. V., Mahamuni N. M., Pandit A. B. (2016). J. Environ. Manage..

[cit2] Dong S., Feng J., Fan M., Pi Y., Hu L., Han X., Liu M., Sun J., Sun J. (2015). RSC Adv..

[cit3] Bethi B., Sonawane S. H., Bhanvase B. A., Gumfekar S. P. (2016). Chem. Eng. Process. Process Intensif..

[cit4] Reddy P. A. K., Reddy P. V. L., Kwon E., Kim K.-H., Akter T., Kalagara S. (2016). Environ. Int..

[cit5] Khaki M. R. D., Shafeeyan M. S., Raman A. A. A., Daud W. M. A. W. (2017). J. Environ. Manage..

[cit6] Kumar S. G., Rao K. S. R. K. (2017). Appl. Surf. Sci..

[cit7] Han D., Liu J., Cai H., Zhou X., Kong L., Wang J., Shi H., Guo Q., Fan X. (2018). Appl. Surf. Sci..

[cit8] Zhao T., Zai J., Xu M., Zou Q., Su Y., Wang K., Qian X. (2011). CrystEngComm.

[cit9] Yang J., Jiang P., Yue M., Yang D., Cong R., Gao W., Yang T. (2017). J. Catal..

[cit10] Chi F., Song B., Yang B., Lv Y., Ran S., Huo Q. (2015). RSC Adv..

[cit11] Cho S., Lee I.-J., Jung D. (2013). Solid State Sci..

[cit12] Su B., Xie H., Tan Y., Chai S., He Y., Zhang S. (2018). J. Mater. Sci.: Mater. Electron..

[cit13] Radosavljevic J. A. K., Howard, Sleight A. W. (2000). Int. J. Inorg. Mater..

[cit14] Hao S.-Z., Zhou D., Li W.-B., Pang L.-X. (2017). J. Electron. Mater..

[cit15] Barros R., Deloncle J., Deschamp P., Boutinaud G., Chadeyron R., Mahiou E., Cavalli M., Brik G. (2014). Opt. Mater..

[cit16] Evans R., Howard J. A. K., Sleight A. W. (2005). Solid State Sci..

[cit17] Nunes S. E., Wang C.-H., So K., Evans J. S. O., Evans I. R. (2015). J. Solid State Chem..

[cit18] Liu H., Imanishi A., Yang W., Nakato Y. (2010). Electrochim. Acta.

[cit19] Liu H., Nakamura R., Nakato Y. (2006). Electrochem. Solid-State Lett..

[cit20] Luo H., Li J., Xu J., Fang L., Tang Y., Li C. (2016). J. Mater. Sci.: Mater. Electron..

[cit21] Banerjee S., Pillai S. C., Falaras P., O'shea K. E., Byrne J. A., Dionysiou D. D. (2014). J. Phys. Chem. Lett..

[cit22] Kou J., Lu C., Wang J., Chen Y., Xu Z., Varma R. S. (2017). Chem. Rev..

[cit23] Miyazaki K., Sato H., Kikuchi S., Nakatani H. (2014). J. Appl. Polym. Sci..

[cit24] Zhang C. F., Qiu L. G., Ke F., Zhu Y. J., Yuan Y. P., Xu G. S., Jiang X. (2013). J. Mater. Chem. A.

[cit25] Chang H., Jo E. H., Jang H. D., Kim T. O. (2013). Mater. Lett..

[cit26] Moradi S., Vossoughi M., Feilizadeh M., Zakeri S. M. E., Mohammadi M. M., Rashtchian D., Booshehri A. Y. (2015). Res. Chem. Intermed..

[cit27] Nawawi W. I., Zaharudin R., Zuliahani A., Shukri D. S., Azis T. F., Razali Z. (2017). Appl. Sci..

[cit28] Zhang J., Zhang P., Ma K., Han F., Chen G., Wei X. (2008). Sci. China, Ser. B: Chem..

The article "Polyethylene glycol-doped BiZn2VO6 as a high-efficiency solar-light-activated photocatalyst with substantial durability toward photodegradation of organic contaminations" was retracted in 2023. Reasons: an official misconduct investigation; misconduct by an author.

[cit29] Wong K. W., Field M. R., Ou J. Z., Latham K., Spencer M. J., Yarovsky I., Kalantar-zadeh K. (2011). Nanotechnology.

[cit30] Kamiura Y., Yamashita Y., Nakamura S. (1998). Jpn. J. Appl. Phys..

[cit31] Reunchan P., Umezawa N. (2013). Phys. Rev. B.

[cit32] Elhag S., Tordera D., Deydier T., Lu J., Liu X., Khranovskyy V., Hultman L., Willander M., Jonsson M. P., Nur O. (2017). J. Mater. Chem. A.

[cit33] Cooper J. K., Scott S. B., Ling Y., Yang J., Hao S., Li Y., Toma F. M., Stutzmann M., Lakshmi K. V., Sharp I. D. (2016). Chem. Mater..

[cit34] Hu X., Zhu Q., Gu Z., Zhang N., Liu N., Stanislaus M. S., Li D., Yang Y. (2017). Ultrason. Sonochem..

[cit35] Liu X., Zhong J., Li J., Huang S., Song W. (2015). Appl. Phys. A.

[cit36] Van de Walle C. G. (2000). Phys. Rev. Lett..

[cit37] Qiu J., Dawood J., Zhang S. (2014). Chin. Sci. Bull..

[cit38] Lorite I., Wasik J., Michalsky T., Schmidt-Grund R., Esquinazi P. (2014). Thin Solid Films.

[cit39] Park S., Mun Y., An S., Lee W. I., Lee C. (2014). J. Lumin..

[cit40] Tsiarapas C., Girginoudi D., Georgoulas N. (2014). Semicond. Sci. Technol..

[cit41] Limpijumnong S., Zhang S. B. (2005). Appl. Phys. Lett..

[cit42] Lavrov E. V., Weber J. (2006). Phys. Rev. B.

[cit43] Lavrov E. V., Börrnert F., Weber J. (2005). Phy. Rev. B.

[cit44] Elhag S., Khun K., Khranovskyy V., Liu X., Willander M., Nur O. (2016). Sensors.

[cit45] Liu J., Lu W., Zhong Q., Jin X., Wei L., Wu H., Zhang X., Li L., Wang Z. (2017). Mol. Catal..

[cit46] Fatima S., Ali S. I., Iqbal M. Z., Rizwan S. (2017). RSC Adv..

[cit47] Xin Z., Li L., Zhang X., Zhang W. (2018). RSC Adv..

[cit48] Anandan M., Dinesh S., Krishnakumar N., Balamurugan K. (2016). J. Mater. Sci.: Mater. Electron..

[cit49] Chen R., Zhu C., Lu J., Xiao J., Lei Y., Yu Z. (2018). Appl. Surf. Sci..

[cit50] Bosacka M., Kurzawa M., Rychlowska-Himmel I., Szkoda I. (2005). Thermochim. Acta.

[cit51] Zhang L., Yan J., Zhou M., Yang Y., Liu Y.-N. (2013). Appl. Surf. Sci..

[cit52] Feng C., Wang D., Jin B., Jiao Z. (2015). RSC Adv..

[cit53] Cai P., Zhou S.-M., Ma D.-K., Liu S.-N., Chen W., Huang S.-M. (2015). Nano-Micro Lett..

[cit54] Shan L.-W., Wang G.-L., Suriyaprakash J., Li D., Liu L.-Z., Dong L.-M. (2015). J. Alloys Compd..

[cit55] Bora L. V., Mewada R. K. (2017). Renewable Sustainable Energy Rev..

[cit56] Zheng W., Ding R., Yan X., He G. (2017). Mater. Lett..

[cit57] Ko F.-H., Lo W.-J., Chang Y.-C., Guo J.-Y., Chen C.-M. (2016). J. Alloys Compd..

[cit58] Khranovskyy V., Lazorenko V., Lashkarev G., Yakimova R. (2012). J. Lumin..

[cit59] Chang Y.-C. (2014). J. Alloys Compd..

[cit60] Malara F., Fabbri F., Marelli M., Naldoni A. (2016). ACS Catal..

[cit61] Zhang J. Z., Yan Y. (2018). J. Taiwan Inst. Chem. Eng..

The article "Polyethylene glycol-doped BiZn2VO6 as a high-efficiency solar-light-activated photocatalyst with substantial durability toward photodegradation of organic contaminations" was retracted in 2023. Reasons: an official misconduct investigation; misconduct by an author.

[cit62] Li P., Chen Q., Lin Y., Chang G., He Y. (2016). J. Alloys Compd..

[cit63] Aghabeygi S., Khademi-Shamami M. (2018). Ultrason. Sonochem..

[cit64] Kumar N., Sen A., Rajendran K., Rameshbabu R., Ragupathi J., Therese H. A., Maiyalagan T. (2017). RSC Adv..

[cit65] Chaudhary A., Mohammad A., Mobin S. M. (2018). Mater. Sci. Eng., B.

[cit66] Shambharkar B. H., Chowdhury A. P. (2018). J. Environ Chem. Eng..

[cit67] Liu A.-L., Li Z.-Q., Wu Z.-Q., Xia X.-H. (2018). Talanta.

[cit68] Herrmann J. M. (1999). Catal. Today.

[cit69] Gao L., Gan W., Qiu Z., Zhan X., Qiang T., Li J. (2017). Sci. Rep..

[cit70] Mousavi M., Habibi-Yangjeh A., Pouran S. R. (2018). J. Mater. Sci.: Mater. Electron..

[cit71] Cooper J. K., Scott S. B., Ling Y., Yang J., Hao S., Li Y., Toma F. M., Stutzmann M., Lakshmi K. V., Sharp I. D. (2016). Chem. Mater..

[cit72] Wang G., Ling Y., Lu X., Qian F., Tong Y., Zhang J. Z., Lordi V., Rocha Leao C., Li Y. (2013). J. Phys. Chem. C.

[cit73] Pirhashemi M., Habibi-Yangjeh A., Pouran S. R. (2018). J. Ind. Eng. Chem..

[cit74] Kanagaraj T., Thiripuranthagan S., Paskalis S. M. K., Abe H. (2017). Appl. Surf. Sci..

[cit75] Yang Z., Ding J., Feng J., He C., Li Y., Tong X., Niu X., Zhang H. (2018). Appl. Organomet. Chem..

[cit76] Huang Y., Li K., Lin Y., Tong Y., Liu H. (2018). ChemCatChem.

[cit77] Liu P., Sun H., Liu X., Sui H., Zhang Y., Zhou D., Guo Q., Ruan Y. (2017). J. Am. Ceram. Soc..

[cit78] Li S., Hu S., Jiang W., Liu Y., Zhou Y., Liu J., Wang Z. (2018). J. Colloid Interface Sci..

[cit79] Cui Y., Zhang X., Guo R., Zhang H., Li B., Xie M., Cheng Q., Cheng X. (2018). Sep. Purif. Technol..

[cit80] Wang Y., Sunarso J., Zhao B., Ge C., Chen G. (2017). Ceram. Int..

[cit81] Yuan H., Lunt R. R., Blanchard G. J., Ofoli R. Y. (2016). ChemElectroChem.

[cit82] Wang A., Zhang J., Zhao W., Zhu W., Zhong Q. (2018). J. Alloys Compd..

[cit83] Xu Y., Lin D., Liu X., Luo Y., Xue H., Huang B., Chen Q., Qian Q. (2018). ChemCatChem.

[cit84] Liu X., Zhong J., Li J., Huang S., Song W. (2015). Appl. Phys. A.

[cit85] Ghalajkhani A., Haghighi M., Shabani M. (2018). J. Photochem. Photobiol., A.

